The article "Habitat and introduced predators influence the occupancy of small threatened macropods in subtropical Australia" was published in 2019. Journal: Ecol Evol.

# Habitat and introduced predators influence the occupancy of small threatened macropods in subtropical Australia

**DOI:** 10.1002/ece3.5203

**Published:** 2019-04-29

**Authors:** Darren McHugh, Ross L. Goldingay, Jeremy Link, Mike Letnic

**Affiliations:** ^1^ School of Environment, Science and Engineering Southern Cross University Lismore New South Wales Australia; ^2^ NSW National Parks and Wildlife Service Iluka New South Wales Australia; ^3^ Centre for Ecosystem Science, School of Biological, Earth and Environmental Sciences University of New South Wales Sydney New South Wales Australia

**Keywords:** dingo, habitat, long‐nosed potoroo, mesopredator, occupancy modeling, red‐legged pademelon

## Abstract

Australia has had the highest rate of mammal extinctions in the past two centuries when compared to other continents. Frequently cited threats include habitat loss and fragmentation, changed fire regimes and the impact of introduced predators, namely the red fox (*Vulpes vulpes*) and the feral cat (*Felis catus*). Recent studies suggest that Australia's top predator, the dingo (*Canis dingo*), may have a suppressive effect on fox populations but not on cat populations. The landscape of fear hypothesis proposes that habitat used by prey species comprises high to low risk patches for foraging as determined by the presence and ubiquity of predators within the ecosystem. This results in a landscape of risky versus safe areas for prey species. We investigated the influence of habitat and its interaction with predatory mammals on the occupancy of medium‐sized mammals with a focus on threatened macropodid marsupials (the long‐nosed potoroo [*Potorous tridactylous*] and red‐legged pademelon [*Thylogale stigmatica*]). We assumed that differential use of habitats would reflect trade‐offs between food and safety. We predicted that medium‐sized mammals would prefer habitats for foraging that reduce the risk of predation but that predators would have a positive relationship with medium‐sized mammals. We variously used data from 298 camera trap sites across nine conservation reserves in subtropical Australia. Both dingoes and feral cats were broadly distributed, whilst the red fox was rare. Long‐nosed potoroos had a strong positive association with dense ground cover, consistent with using habitat complexity to escape predation. Red‐legged pademelons showed a preference for open ground cover, consistent with a reliance on rapid bounding to escape predation. Dingoes preferred areas of open ground cover whereas feral cats showed no specific habitat preference. Dingoes were positively associated with long‐nosed potoroos whilst feral cats were positively associated with red‐legged pademelons. Our study highlights the importance of habitat structure to these threatened mammals and also the need for more detailed study of their interactions with their predators.

The article "Habitat and introduced predators influence the occupancy of small threatened macropods in subtropical Australia" was published in 2019. Journal: Ecol Evol.

## 1 INTRODUCTION

The terrestrial mammal fauna of Australia has suffered an extinction loss disproportional to that of other nations during the past two centuries (Fisher et al., 2014; Johnson, Isaac, & Fisher, 2007; Short & Smith, 1994; Woinarski, Burbidge, & Harrison, 2015). Thirty terrestrial mammal species have become extinct in Australia in the past 200 years representing 11% of Australia's mostly endemic terrestrial mammal species (Woinarski et al., 2015). At present, there are 30 terrestrial mammal species listed as endangered and 46 species listed as vulnerable under Australian federal legislation: *Environment Protection & Biodiversity Conservation Act 1999*. Medium‐sized mammals (body mass 0.5–5.5 kg) have incurred more losses and declines than small‐sized mammals (Burbidge & McKenzie, 1989; Cardillo & Bromham, 2001; Johnson & Isaac, 2009). In order to provide effective conservation for threatened medium‐sized mammals, it is important to determine the factors that influence or limit their occurrence.

Frequently cited threats to Australia's medium‐sized mammals include habitat loss and fragmentation (Bennet, 1990; Law & Dickman, 1998; Lindenmayer, McCarthy, Parris, & Pope, 2000; McAlpine & Eyre, 2002; McAlpine et al., 2006), inappropriate fire regimes (Hradsky, Mildwaters, Ritchie, Christie, & Stefano, 2017), weed invasion (e.g., *lantana camara* (Turner & Downey, 2010)) and predation by introduced predators; the red fox (*Vulpes vulpes*) and feral cat (*Felis catus*) (Doherty et al., 2015; Kinnear, Onus, & Bromilow, 1988; Kinnear, Sumner, & Onus, 2002; Radford et al., 2018; Short & Smith, 1994). The impacts of introduced predators may have been exacerbated in some areas by the suppression of dingo (*Canis dingo*) populations, as dingoes have a suppressive effect on the abundances of foxes and cats in some ecosystems (Kennedy, Phillips, Legge, Murphey, & Faulkner, 2011; Leo, Reading, Gordon, & Letnic, 2018; Letnic et al., 2011). Consequently, where dingoes have been removed the abundances of introduced predators and their impacts on medium‐sized mammals tend to increase (Johnson et al., 2007).

The structure and quality of habitat exert a strong influence over the occurrence and movement of ground‐dwelling mammals (Catling & Burt, 1995). Many medium‐sized mammals require a range of understory habitats to fulfill important biological functions, for example, obtain food, water, to find potential mates and to provide shelter from predators and the elements at both daily and seasonal temporal scales (Creel, Winnie, Maxwell, Hamlin, & Creel, 2005; Kauffman et al., 2007). For example, the presence of physically complex understory vegetation provides nocturnal medium‐sized mammals with important diurnal nesting sites (Norton, Prentice, Dingle, French, & Claridge, 2015) whereas adjoining areas of open understory are required to forage in at night (Vernes, 1995). Over longer temporal gradients, many ground‐dwelling mammals require multiple habitats to obtain resources as they become available in different locations (Law & Dickman, 1998). The landscape of fear (LoF) hypothesis proposes that the habitat available to prey species comprises high to low risk patches due to spatial heterogeneity in the threat posed by predators (Laundré et al., 2014; Shrader, Brown, Kerley, & Kotler, 2008). Thus, prey individuals may avoid or minimize the time they spend in habitats where the perceived risk of predation is high (Brown & Kotler, 2004; Laundré et al., 2014). For example, many studies have shown that small mammals display a strong preference for densely vegetated habitats which provide shelter from predators (Brown & Kotler, 2004). Therefore, habitat use should not be viewed simply from the perspective of foraging success but should include consideration of trade‐offs imposed by predation risk.

The article "Habitat and introduced predators influence the occupancy of small threatened macropods in subtropical Australia" was published in 2019. Journal: Ecol Evol.

Simplification of understory habitats due to grazing by large introduced herbivores and inappropriate fire regimes is thought to exacerbate the impacts that introduced predators have on native mammals (Hradsky et al., 2017). However, few studies have focused on predator–prey relationships in subtropical Australia where topography and habitat structure are complex, yet this is where many of these mammals continue to persist (Reside et al., 2013). Given the importance of habitat structural complexity, management of habitat has proven to be critical for the persistence of some threatened species (Lawes et al., 2015).

The mesic forests of eastern Australia are important refugia for several threatened and common medium‐sized mammals (Reside et al., 2013), which have declined in other regions. For example, the threatened long‐nosed potoroo (*Potorous tridactylus*) has suffered a major range contraction on the coastal plains of northern New South Wales (NSW), Australia, due to increased development that has resulted in the loss of large areas of habitat (Andren, Milledge, Scotts, & Smith, 2018). The adjacent ranges within northern NSW have maintained critical habitat for this species in the absence of development pressures.

The mesic forests of eastern Australia appear to function as refugia for potoroos and other ground‐dwelling medium‐sized mammals for several reasons: (a) large areas of mesic forests are protected within conservation areas and therefore are not subject to complete loss of habitat, (b) they provide reliable and relatively sustained food resources, and (c) highly productive areas (high rainfall and soil fertility) result in physically complex habitat structure which help mammals to avoid introduced predators. These forests also provide habitat for dingoes, wild dogs, and their hybrids and perhaps as a consequence the introduced red fox is relatively scarce (Catling & Burt, 1997). Thus, predation by red foxes is thought to have a relatively minor impact on medium‐sized mammals (Johnson & VanDerWal, 2009). It must be noted that there is taxonomic instability and contention regarding the taxonomy of the dingo (see Smith et al., 2019; Jackson et al., 2019). For the purpose of our study, we do not discriminate between dingoes/wild dogs and their hybrids.

The article "Habitat and introduced predators influence the occupancy of small threatened macropods in subtropical Australia" was published in 2019. Journal: Ecol Evol.

The aim of this study was to investigate the influence of habitat and predatory mammals on the occupancy of medium‐sized terrestrial mammals across nine conservation reserves (totaling 89,906 ha) in subtropical eastern Australia where a combination of high rainfall and fertile soils provides a landscape dominated by structurally complex forests (Keith, 2004). We conducted occupancy analysis on data from two camera trapping surveys. We had a particular focus on two threatened marsupials from the superfamily macropodoidea (hereafter macropods); the long‐nosed potoroo and the red‐legged pademelon (*Thylogale stigmatica*). A fundamental goal of our study was to determine where in the landscape these threatened species occur to enable conservation programs to be devised.

## 2 METHODS

### 2.1 Study area

This study was conducted within the North Coast Bioregion NSW (Figure 1). Surveys were conducted within nine National Parks (hereafter reserves): Border Ranges, Nightcap (including part of the connected Whian Whian State Conservation Area), Richmond Range, Mebbin, Mt Jerusalem, Toonumbar, Yabbra, Tooloom, and Koreelah (Figure 1). The study area is dominated by the iconic Tweed shield volcano comprising Mt Warning (Wollumbin) and its surrounding caldera which is known for its significant biodiversity values (Floyd, 1990; Kitching, Braithwaite, & Cavanaugh, 2011). The landscape is characterized by mountain ranges and plateaux of basaltic and rhyolitic origin at higher elevations (500–1,100 m) that support significant stands of World Heritage listed subtropical rainforest (Keith, 2004). At fertile mid‐elevations (300–500 m) with annual rainfall > 1,000 mm, North Coast Wet Sclerophyll forests dominated by flooded gum (*Eucalyptus grandis*), brush box (*Lophostemon confertus*), and tallowwood (*Eucalyptus microcorys*) are present (Keith, 2004). At lower elevations (<300 m), the landscape supports Clarence Dry Sclerophyll forests dominated by spotted gum (*Corymbia variegata*), grey ironbark (*E. siderophloia*), pink bloodwood (*C. intermedia*), and grey gum (*E. propinqua*) (Keith, 2004). The region experiences a humid subtropical climate with an average annual rainfall of 1,247 mm (Mean Annual rainfall at Lismore Airport AWS). A marked wet season occurs with summer maximum and winter minimum rainfall. Temperatures are mild to warm all year round with average temperatures of 17.4°C to 29.3°C in summer and 7.3°C to 20.5°C in winter (Australian Bureau of Meteorology Climate Data).

The article "Habitat and introduced predators influence the occupancy of small threatened macropods in subtropical Australia" was published in 2019. Journal: Ecol Evol.

**Figure 1:** Study area and monitoring sites within nine national parks (NP) of the north coast bioregion of northern New South Wales, Australia. Numbers within brackets indicate number of camera traps within each national park

### 2.2 Survey design and camera trapping

Camera trap sites were established broadly throughout each reserve in linear transects along access roads and management trails to maximize coverage over each reserve (Figure 1). We established 298 sites with the number in each reserve reflecting its area. Reconyx Rapidfire^™^ HC 500 (infrared flash) and HC550 (white flash) cameras were deployed alternating across the sites, at least 500 m apart. Cameras were positioned within 50 m of track and management trail edges. We considered this distance was a suitable compromise to maximize detection of predators which frequent areas on and close to roads (Meek, Ballard, Fleming, & Falzon, 2016) and medium‐sized mammals which are likely to prefer vegetative cover (MacQueen, Seddon, & Goldizen, 2011; Norton et al., 2015). The distance between sites was selected based on the home ranges of two of the threatened medium‐sized mammals we expected to detect, the long‐nosed potoroo and red‐legged pademelon. These species have home ranges < 6 ha in area (Long, 2001; Vernes, 1995). If these home ranges are approximately circular, their diameter would be <280 m.

Each camera was fixed to a tree at a height of 40 cm, directed at a wooden stake (40 cm high) at approximately 2.5 m from the camera. All obstructing vegetation between the camera and lure station was removed. A perforated PVC pipe (5 × 15 cm) was fixed to each stake to hold one of two lure types. A mix of peanut butter and oats was used to attract native ground‐dwelling mammals and a combination of chicken neck and tuna oil was used to attract predators (Robley et al., 2014). These lure types were randomized across site locations.

The article "Habitat and introduced predators influence the occupancy of small threatened macropods in subtropical Australia" was published in 2019. Journal: Ecol Evol.

Cameras operated 24 hr per day for a duration of 21 days (3 weeks) during each monitoring period and were set to take five images per trigger (one picture per second) with a quiet time between triggers of one minute. The 21‐day period was influenced by previous camera trapping of potoroos, pademelons, and bandicoots in Richmond Range which showed that a 3‐week period gave a 95% probability of detection of these species (Taylor, Goldingay, & Lindsay, 2014).

Each camera was set for medium/high sensitivity and recorded the time, date, and ambient temperature. Cameras were deployed in two monitoring periods across each of the nine reserves. Only 2–3 reserves could be monitored concurrently with the remaining reserves monitored consecutively. Period one occurred between May and August 2016, and period two occurred between October 2016 and January 2017.

### 2.3 Habitat assessments

Habitat assessments were undertaken along two 25 m transects centered at each camera monitoring site and orientated north‐south and east‐west. Measures of cover were taken at 1‐m intervals along each transect. A 20 × 50 cm chequered coverboard was used to record ground cover was measured within 0–0.5 m from the ground and shrub cover 1–1.5 m above ground. A cross‐hair was used to record the presence/absence of canopy cover. The 50 records of each measure were used to produce an overall percentage. The vegetation at each site was recorded as subtropical rainforest or sclerophyll eucalypt forest.

### 2.4 Testing of hypotheses

We tested a set of hypotheses relating to habitat preferences for the medium‐sized mammals, and predator–prey relationships based on dietary studies for dingoes and feral cats (Table 1). These hypotheses are a manifestation of the landscape of fear hypothesis that relate to our target species at the regional scale. For the threatened macropods, we predicted that they would only occur across a subset of conservation reserves whereas other species should be widespread across most conservation reserves. The long‐nosed potoroo is well documented to be in decline in our region (Andren, Milledge, Scotts, & Smith, 2013). We hypothesized that ground cover and shrub cover are likely to have a positive influence over long‐nosed potoroo and bandicoot occupancy. We have assumed that the different categories of these microhabitats do not vary in food availability but any differential use reflects the trade‐off made with predation risk. These species show a preference toward dense habitats that may provide concealment from predators (Claridge & Barry, 2000; Norton, French, & Claridge, 2011). We hypothesized that vegetation type (rainforest or eucalypt forest) would be influential over both red‐legged and red‐necked pademelon occupancy because these species are documented to show a preference for rainforest habitat types (Johnson & Vernes, 1994; Wahungu, Catterall, & Olsen, 2001).

The article "Habitat and introduced predators influence the occupancy of small threatened macropods in subtropical Australia" was published in 2019. Journal: Ecol Evol.

**Table 1:** Hypotheses that may explain the influence of habitat covariates (a) or species interactions (b) on occupancy by medium‐sized mammals, and their mammalian predators

Species	Hypothesis	Covariates	References
(a) Habitat & Reserve covariates	red‐legged pademelons and potoroos persist in a subset of reserves due to restricted distributions	Reserve	Andren et al. (2013)
	Red‐legged and red‐necked pademelons show a preference for open areas in rainforest vegetation	Vegetation	Vernes (1995)
	Potoroos and bandicoots favor dense habitats that provide concealment from predators	Ground & shrub cover	Catling and Barry (2000), Norton et al. (2015)
	Dingoes/wild dogs are widespread	Reserve	Catling and Burt (1995)
	Feral cats are widespread	Reserve	Catling and Burt (1995)
(b) Species interactions	The occupancy of the feral cat is independent of the dingo	Feral Cat	Wang and Fisher (2012), Brook et al. (2012)
	Dingo occurrence aligns with medium‐sized mammals which comprise a large part of their prey	Bandicoots, potoroos, and pademelons	Barker et al. (1994), Glen et al. (2006), and Doherty et al. (2018)
	Cat occurrence aligns with Medium‐sized mammals which are considered prey species	Bandicoots, potoroos, and pademelons	Scott (1994), Lazenby (2012), and Fancourt (2015)

Previous studies suggest that red foxes occur in very low densities across the reserves in northern NSW, whilst dingoes and feral cats are broadly distributed (Catling & Burt, 1997). We assumed this would prevail in our study area so that foxes would be rare whereas dingoes and feral cats would have widespread occupancy. We expected to detect a negative relationship between dingoes and foxes (Johnson & VanDerWal, 2009; Letnic et al., 2011). Indeed, we detected the red fox at only seven sites so further analysis was not possible. We predicted there would be a negligible relationship between dingoes and cats (Allen, Engeman, & Leung, 2015; Brook, Johnson, & Ritchie, 2012; Wang & Fisher, 2012). We hypothesized that predators were likely to be influential over the probability of detecting their potential prey in accordance with their preferred prey weight ranges. Although dingoes show a preference for larger macropod species in drier regions, in the mesic forests of northern NSW and northern QLD, medium‐sized mammals make up a large portion of their diet (Barker, Lunney, & Bubela, 1994; Doherty et al., 2018; Vernes, Dennis, & Winter, 2001). Therefore, we hypothesized that dingoes would have a positive spatio‐temporal relationship with pademelons, bandicoots, and potoroos. Feral cats are capable of preying on medium‐sized mammals, with bandicoots and long‐nosed potoroos making up a significant portion of their diet at some locations (Lazenby, 2012; Scott, 1994). Also, there is direct evidence that feral cats prey on Tasmanian pademelons (*Thylogale billardierii*) (Fancourt, 2015), therefore we suspect that cats may prey on red‐necked (*Thylogale thetis*) and red‐legged pademelons in our study sites. We hypothesized that feral cats would have a positive spatio‐temporal relationship with these species.

The article "Habitat and introduced predators influence the occupancy of small threatened macropods in subtropical Australia" was published in 2019. Journal: Ecol Evol.

### 2.5 Single‐species occupancy modeling

We aimed to examine the influence of site and survey covariates on detection (P) and occupancy (ψ) for a suite of terrestrial mammal species using single‐season occupancy models in program PRESENCE version 9.3 (USGS Patuxent Wildlife Research Centre). Species included the Federally listed long‐nosed potoroo, the NSW‐listed red‐legged pademelon, the red‐necked pademelon, the long‐nosed bandicoot (*Perameles nasuta*), and the northern brown bandicoot (*Isoodon macrourus*) (hereafter pooled as “bandicoot”), the dingo/wild dog and their hybrids (hereafter dingo) and the feral cat (Figure 2). We also detected the red fox, the NSW‐listed black‐striped wallaby (*Macropus dorsalis*), and the tiger quoll (*Dasyurus maculatus*), but they were detected at too few sites to include in the modeling. The two pademelon species could be readily distinguished due to the pronounced facial stripe, lack of neck shading, presence of leg color and leg stripe in the red‐legged pademelon (Figure 2). Many of the images we obtained were in color. We excluded records in a few instances where animals were obscured. We constructed weekly detection histories across the two 3‐week periods for each species representing whether they were detected (1) or not (0) or if a site was not surveyed or a camera malfunctioned (−).

**Figure 2:** Images of ground‐dwelling mammal species detected in this study: (a) Red‐legged pademelon, (b) Long‐nosed potoroo, (c) Black‐striped wallaby, (d) red‐necked pademelon, (e) Northern Brown bandicoot, (f) northern mountain possum, (g) dingo, (h) red fox, (i) feral cat, and (j) tiger quoll

Occupancy models were constructed to test our set of hypotheses (Table 1). Modeling followed a 2‐step procedure. We started by examining the fit of models on the probability of detection. The detection parameter could be constant or time‐varying (fully or seasonal). We then retained the top model or one in which the probability of detection was constant and examined the influence of site covariates on the probability of occupancy. Models were ranked from lowest to highest AIC (Akaike's Information Criterion). The difference in AIC (∆AIC) between each model and the top model was calculated and was the basis of inferring the plausibility of each model (Burnham & Anderson, 2004). Where ∆AIC was <2 models were considered equally plausible in explaining the data (Burnham & Anderson, 2004). Where ∆AIC was 4–7, the models with the higher AIC were viewed as having less support. If adding an additional covariate to a top model did not reduce AIC by >2, then the covariate was deemed an uninformative parameter and omitted (see Arnold, 2010).

The article "Habitat and introduced predators influence the occupancy of small threatened macropods in subtropical Australia" was published in 2019. Journal: Ecol Evol.

The site covariates include the habitat variables; (a) ground cover, (b) shrub cover, (c) canopy cover, (d) vegetation type, and a variable for individual conservation reserve. To investigate the influence of conservation reserve, we constructed dummy variables (1, 0) for each reserve. Initial models allowed occupancy to be estimated uniquely for each reserve. Competing models were then run with reduced numbers of reserves estimated individually by grouping reserves with similar estimates. We conducted preliminary modeling to investigate whether camera type (white flash or infrared) and lure type (peanut butter and oats or meat) influenced our data. These variables were fixed for the duration of a round of surveys at a site so were included as site covariates. However, due to the way our surveys were done there were some sites (~33%) where the type changed from one survey round to the next. We scored these sites as absent records, to allow the remaining sites to be compared. We found that for all of our targeted species, models with camera and lure type had less support than ones where occupancy was modeled as constant across sites.

Four additional covariates were investigated as part of a preliminary analysis for the dingo. These covariates relate to lethal baiting with 1,080 (sodium fluoroacetate) that have taken place biannually for at least the past five years within five of the nine conservation reserves. We investigated these additional covariates for the dingo because they are plausible factors that may affect/influence dingo occupancy. Baiting of dingoes, wild dogs, and their hybrids is required on Schedule 2 lands (public land that is controlled land) under the *Local Land Service Act 2013* and the *Local Land Services (Wild Dog) pest control order 2015* to minimize the loss of livestock on properties adjoining the reserves. Dingo baiting covariates included whether a reserve was baited (Nightcap NP, Richmond Range NP, Mebbin NP, and Mt Jerusalem NP) or not (Border Ranges NP, Toonumbar NP, Yabbra NP, Tooloom NP, and Koreelah NP), as well as three covariates that were derived from the timing and location of baiting (distance of camera sites to baiting stations, the time interval between baiting and monitoring, and the density of bait stations within a 2 km radius of each camera site). The latter three variables were highly correlated (>0.7) so we only baiting density was investigated. Preliminary analysis revealed that neither reserve baiting status nor baiting density influenced dingo occupancy in a consistent way and performed poorly compared to other site covariates. We presume that this was due to the nature of baiting within reserves which could be considered low intensity and also baiting that occurs within the landscape that could not be accounted for. These results are not reported further.

The article "Habitat and introduced predators influence the occupancy of small threatened macropods in subtropical Australia" was published in 2019. Journal: Ecol Evol.

We assessed model fit of the most parameterized model to the survey data for each species within presence with 10,000 bootstrap samples. This revealed there was no significant lack of fit in the data for the long‐nosed potoroo (*p* = 0.34, c‐hat = 1.04), bandicoots (*p* = 0.40, c‐hat = 0.95), dingo (*p* = 0.86, c‐hat = 0.14), or feral cats (*p* = 0.35, c‐hat = 0.86). However, there was evidence of overdispersion in the data for the red‐legged pademelon (*p* = 0.007, c‐hat = 1.63) and red‐necked pademelon (*p* = 0.01, c‐hat = 2.39). Therefore, we used the c‐hat values to adjust for overdispersion which led to comparison of models using quasi‐AIC (QAIC) (Burnham & Anderson, 2004).

### 2.6 Co‐occurrence occupancy modeling

We investigated interactive effects between pairs of species through the 2‐species occupancy approach of MacKenzie, Bailey, and Nichols (2004). Pairs of species included the dingo with all other medium‐sized mammals separately, the feral cat with all medium‐sized mammals separately and the dingo and feral cat. We used the formulation of Richmond, Hines, and Beissinger (2010) as implemented within presence. This model estimates interaction between two species in occupancy and detection parameters. It estimates the probability of occupancy of one focal species referred to as species A (psi^A^), and a second species referred to as species B. For species B, psi is estimated conditioned on whether species A is present (psi^B/A^) or absent (psi^B/a^). The formulation estimates detection probabilities of each species when the other is absent (*p* ^A^, *p* ^B^) and when the other is present and detected (*r* ^A^, *r* ^B/A^), and for species B, when species A is present but not detected (*r* ^B/a^).

We conducted this modeling by first fitting models to investigate influences on occupancy and then by investigating influences on detection with the top occupancy model retained. For occupancy, we explored two hypotheses: (a) whether species B occurred at sites independently of species A (comparing a model with psi^B/A^ and psi^B/a^ estimated separately with one where psi^B/A^=psi^B/a^), and (b) whether adding a habitat covariate provided a better fit to the best model from (a). We then investigated the detection parameters following the suggestion of MacKenzie et al. (2018). We compared a model with all detection parameters estimated separately (*p* ^A^, *p* ^B^, *r* ^A^, *r* ^B/A^, *r* ^B/a^) with models in which some of these parameters were equal or not equal. We compared detection of species B when species A was present and detected (*r* ^B/A^) to when it was present and not detected (*r* ^B/a^), that is, does (*r* ^B/A ^= *r* ^B/a^). We also tested whether the detection of species B at a site where only it occurred differed to a site where species A also occurred and was detected or not (*p* ^B ^= *r* ^B/A ^= *r* ^B/a^). Another focusing on species A whether species B was detected or not (*p* ^A ^= *r* ^A^), one with both included (*p* ^A ^= *r* ^A^, *p* ^B ^= *r* ^B/a^), and where detection of species B was equal if species A was present or not. Models were compared using AIC as explained above.

The article "Habitat and introduced predators influence the occupancy of small threatened macropods in subtropical Australia" was published in 2019. Journal: Ecol Evol.

## 3 RESULTS

### 3.1 Single‐species, single‐season occupancy models

#### 3.1.1 Long‐nosed potoroo

Long‐nosed potoroos were detected at 33 sites across five reserves: Border Ranges (BR) (*n* = 15), Richmond Range (RR) (*n* = 5), Nightcap (N) (*n* = 5), Tooloom (To) (*n* = 6), and Toonumbar (T) (*n* = 2). The reserves where they were not detected were excluded from the occupancy modeling because it is unknown whether the species has become locally extinct in those reserves. Including these reserves could mean including large numbers of sites where the species simply did not occur. Heterogeneity in detection probability arising from variation in abundance is a concern in occupancy modeling but is expected to be most severe when sampled populations are small (MacKenzie et al., 2018). This will lead to bias in the occupancy estimates. We believe that excluding those reserves should produce more reliable occupancy estimates. The best detection model was one that included “survey round” (model wt = 0.56) (see Table 2 for estimates). This differed to the time‐varying model (wt = 0.38) by ∆AIC 0.79 and from the null model by ∆AIC 4.64 (wt = 0.06). Survey round was included in the modeling of all site covariates. The highest ranked occupancy model was one that included ground cover and where reserves were partitioned into three groups (BR vs. RR = NC = To vs. T) (wt = 0.83). The probability of long‐nosed potoroo occupancy was highest (0.75 ± 0.13) in the Border Ranges in the densest ground cover class (71%–100%), and lowest (0.049 ± 0.04) in Toonumbar within the lowest ground cover class (0%–30%) (Figure 3).

The article "Habitat and introduced predators influence the occupancy of small threatened macropods in subtropical Australia" was published in 2019. Journal: Ecol Evol.

**Table 2:** Naïve occupancy and estimates of the probability of detection

Species	Naïve occupancy	Detection probability	
		Season 1	Season 2
Long‐nosed potoroo	0.18	0.26 ± 0.05	0.13 ± 0.03
Red‐legged pademelon	0.43	0.23 ± 0.02	0.39 ± 0.02
Red‐necked pademelon	0.16	0.31 ± 0.05	0.20 ± 0.04
Bandicoots	0.26	0.21 ± 0.03	
Dingo	0.18	0.14 ± 0.03	
Feral cat	0.17	0.11 ± 0.03	

Note

Only a single detection value is shown where the top detection model included detection as constant across seasons.

**Figure 3:** The probability of occupancy for long‐nosed potoroos, bandicoots, red‐legged pademelons, red‐necked pademelons, dingoes, and feral cats with covariates that were most influential over these species. Percentage of ground cover (0–50 cm) categories (0%–30%, 31%–50%, 51%–70% and 71%–100%) are denoted on the *x* axis for species where it was influential over occupancy. Reserves are denoted on *x* axis by letters or by name and some are shown as groups (=) in some models where occupancy was estimated as equal. BR, Border Ranges; K, Koreelah; M, Mebbin; NC, Nightcap; RR, Richmond Range; T, Toonumbar; To, Tooloom; Y, Yabbra

#### 3.1.2 Bandicoots

Bandicoots were detected at 78 sites: Border Ranges (*n* = 15), Koreelah (K) (*n* = 6), Mebbin (M) (*n* = 11), Nightcap (*n* = 13), Richmond Range (*n* = 5), Tooloom (*n* = 10), Toonumbar (*n* = 9), and Yabbra (Y) (*n* = 9). They were not detected in Mt Jerusalem (MtJ); therefore, this reserve was omitted from analysis. The top detection model was one where bandicoot detection was constant (wt = 0.71) (see Table 2 for estimate). The survey round detection model ranked second (wt = 0.27, ∆AIC = 1.95). The time‐varying model had less support (wt = 0.00, ∆AIC = 8.67). The top occupancy model was where occupancy was estimated for four groups of reserves (M vs. BR = K = NC = To = T = Y vs. RR) (wt = 0.97) (Table 3). Occupancy varied from 0.75 ± 0.16 in Mebbin to 0.23 ± 0.09 in Richmond Range (Figure 3).

**Table 3:** Species occupancy models

Model	AIC	∆AIC	*w*	Model likelihood	*K*
Long‐nosed potoroo					
psi (3 reserve subsets + ground cover), p (survey)	362.40	0.00	0.83	1.00	6
psi (3 reserve subsets), p (survey)	365.46	3.06	0.17	0.22	5
Red‐legged pademelon^a^					
psi (4 reserve subsets + ground cover), p (survey)	730.60	0.00	0.93	1.00	7
psi (4 reserve subsets), p (survey)	733.89	3.29	0.07	0.19	6
Red‐necked pademelon^a^					
psi (2 reserve subsets), p (survey)	196.84	0.00	0.99	1.00	4
psi (8 reserves), p (survey)	207.31	10.47	0.01	0.00	10
Bandicoots					
psi (4 reserve subsets), p (.)	766.43	0.00	0.97	1.00	5
psi (.), p (.)	773.65	7.22	0.03	0.03	10
Dingo					
psi (2 reserve subsets + ground cover), p (.)	531.12	0.00	0.91	1.00	4
psi (2 reserve subsets), p (.)	535.89	4.77	0.08	0.09	3
Feral cat					
psi (2 reserve subsets), p (.)	392.38	0.00	0.95	1.00	3
psi (6 reserves), p (.)	398.36	5.98	0.05	0.05	7

Note

Only the top two models are shown. The number of reserve subsets is the number of grouped reserves where occupancy was uniquely estimated.

(.) = probability of occupancy or detection constant; *K* = number of parameters; *w* = model weight.

a Species where QAIC and ∆QAIC were used.

The article "Habitat and introduced predators influence the occupancy of small threatened macropods in subtropical Australia" was published in 2019. Journal: Ecol Evol.

#### 3.1.3 Red‐legged pademelons

Red‐legged pademelons were detected at 127 sites across all reserves: Border Ranges (*n* = 13), Koreelah (*n* = 4), Mebbin (*n* = 11), Mt Jerusalem (*n* = 1), Nightcap (*n* = 22), Richmond Range (*n* = 25), Tooloom (*n* = 12), Toonumbar (*n* = 20), and Yabbra (*n* = 19). The top detection model was where red‐legged pademelons were influenced by the survey round (wt = 0.95) (see Table 2 for estimates). The full time‐varying model differed to the top model (survey round) by ∆AIC 6.07. The top occupancy model was one which included four groups of reserves (RR, BR = K = To, *M* = NC = T = Y, and MtJ), and ground cover (wt = 0.93) (Table 3). This showed that occupancy decreased from the lowest to highest ground cover class and was highest in Richmond Range and lowest in Mt Jerusalem (Figure 3).

#### 3.1.4 Red‐necked pademelon

Red‐necked pademelons were detected at 43 sites: Border Ranges (*n* = 4), Koreelah (*n* = 2), Mebbin (*n* = 2), Nightcap (*n* = 6), Richmond Range (*n* = 4), Tooloom (*n* = 17), Toonumbar (*n* = 2), and Yabbra (*n* = 6). They were not detected in Mt Jerusalem and therefore this reserve was excluded from further modeling. The top detection model was where detection was influenced by the survey round (wt = 0.71) (see Table 2 for estimates) which was 2.04 ∆AIC above the constant detection model (wt = 0.25). Red‐necked pademelons had a higher probability of detection in the first round (0.31 ± 0.05) compared to the second round (0.20 ± 0.04). There was a strong reserve influence (model wt = 0.99) on the probability of occupancy with Tooloom (0.84 ± 0.14) having a much higher occupancy compared to all other reserves (0.16 ± 0.03) (Figure 3, Table 3).

#### 3.1.5 Dingo

Dingoes were detected at 52 sites across all reserves: Border Ranges (*n* = 6), Koreelah (*n* = 1), Mebbin (*n* = 4), Mt Jerusalem (*n* = 5), Nightcap (*n* = 5), Richmond Range (*n* = 14), Tooloom (*n* = 6), Toonumbar (*n* = 7), and Yabbra (*n* = 4). The top detection model included constant detection (wt = 0.62) (see Table 2 for estimate), which differed to the model with different detection in the two survey rounds ∆AIC of 1.71 (wt = 0.26). The highest ranked occupancy model was one that included ground cover and where reserves were partitioned into two groups (Richmond Range vs. all other reserves) (wt = 0.91). The probability of dingo occupancy varied from 0.94 ± 0.16 in Richmond Range where ground cover was low (0%–30%), to 0.11 ± 0.06 in all other reserves where ground cover was high (71%–100%) (Figure 3).

The article "Habitat and introduced predators influence the occupancy of small threatened macropods in subtropical Australia" was published in 2019. Journal: Ecol Evol.

#### 3.1.6 Feral cat

Feral cats were detected at 39 sites within six reserves: Border Ranges (*n* = 19), Nightcap (*n* = 5), Richmond Range (*n* = 2), Tooloom (*n* = 3), Toonumbar (*n* = 4), and Yabbra (*n* = 6). Feral cats were not detected in Mebbin, Koreelah, or Mt Jerusalem so these reserves were excluded from further modeling for the reasons explained under long‐nosed potoroo above. The top detection model was where detection of feral cats was constant (wt = 0.60) (see Table 2 for estimate). This model differed to one where detection differed in the two survey rounds by ∆AIC = 1.24 (wt = 0.32). No habitat covariates were influential over feral cat occupancy. The top occupancy model was one where the probability of occupancy of feral cats was highest in the Border Ranges versus all other reserves where it was detected (wt = 0.95) (Figure 3).

### 3.2 Two‐species, single‐season occupancy models

#### 3.2.1 Dingo and long‐nosed potoroo

The model with the best support estimated the probability of occupancy of the potoroo and the dingo varied with ground cover (Figure 4). The long‐nosed potoroo favored dense ground cover, with the highest occupancy in dense ground cover areas where the dingo was present (0.78 ± 0.23) compared to dense areas where the dingo was absent (0.48 ± 0.19). Long‐nosed potoroos had the lowest occupancy in open ground cover areas where dingo was absent (0.07 ± 0.05). Dingoes favored areas of open ground cover (0.51 ± 0.09) compared to areas of dense ground cover (0.28 ± 0.11) (Figure 4).

**Figure 4:** Plots of output from co‐occurrence occupancy models where *y* axis shows probability of occupancy and *x* axis shows pairs of species and percentage of ground cover (0–50 cm) categories (0%–30%, 31%–50%, 51%–70%, and 71%–100%). (a) Co‐occurrence of the long‐nosed potoroo and the dingo and dingo probability of occupancy at potoroo sites as a function of ground cover, (b) Co‐occurrence of the red‐legged pademelon and the dingo as a function of ground cover, (c) Co‐occurrence of bandicoots and the dingo as a function of ground cover, and (d) co‐occurrence of the red‐legged pademelon and feral cat

The detection probability of the potoroo varied across the two years. Where dingoes were absent it was estimated at 0.55 ± 0.12 during the first period and 0.02 ± 0.02 during the second period. The top model predicted potoroo detectability as equal when dingoes were present and detected, and present and not detected (*r* ^B/A^ = *r* ^B/a^ = 0.15 ± 0.04). The estimate of phi (species interaction factor) varied with ground cover (0%–30% = 1.67, 95%CI = 1.05–2.30; 31%–50% = 1.70, 95%CI = 1.08–2.31; 51%–70% = 1.59, 95%CI = 0.82–2.36; 71%–100% = 1.39, 95%CI = 0.47–2.30) suggesting that the dingo was influential over potoroo occupancy, particularly in open ground cover habitat (0%–50% cover) where the 95%CIs were >1. The estimate of the detection interaction factor (delta) was 1.0, suggesting detection of one species did not influence the other at sites where they both occurred.

The article "Habitat and introduced predators influence the occupancy of small threatened macropods in subtropical Australia" was published in 2019. Journal: Ecol Evol.

#### 3.2.2 Dingo and red‐legged pademelon

Modeling of the dingo with the red‐legged pademelon revealed that the model with the best support estimated the probability of occupancy of the red‐legged pademelon as equal whether the dingo was present or not (Table 4). Both the dingo and red‐legged pademelon were influenced by ground cover with the dingo having the highest probability of occupancy in open ground cover areas (0.41 ± 0.06) compared to dense ground cover habitat (0.20 ± 0.07) and the red‐legged pademelon probability of occupancy when dingo was present or absent (psi^B/A^ = psi^B/a^) also being higher in open ground cover areas (0.61 ± 0.05) compared to dense ground cover habitat (0.37 ± 0.07) (Figure 4). The detection of the dingo was not dependent on red‐legged pademelons, with dingo detection being equal when red‐legged pademelons were both present or absent (*p* ^A ^= *r* ^A^ = 0.14 ± 0.03). The detection probability of red‐legged pademelons was lower when dingoes were absent (*p* ^B^ = 0.27 ± 0.04) than when dingoes were present with no difference between when dingoes were detected or not (*r* ^B/A ^= *r* ^B/a^ = 0.41 ± 0.05). The estimate of phi was 1.0 suggesting no interaction between these two species. The delta value was also 1.0, suggesting detection of one species did not influence the other.

**Table 4:** Two‐species occupancy models

Model	AIC	∆AIC	*w*	*K*	−2L
Dingo—Long‐nosed potoroo					
psi^A^ (gc)*,* psi^B/A^ (gc), psi^B/a ^(gc),* p* ^A ^= *r* ^A^, *p* ^B^(2)*, r* ^B/A ^= *r* ^B/a^	767.27	0.00	0.98	10	747.27
psi^A^ (gc)*,* psi^B/A^ (gc), psi^B/a ^(gc),* p* ^A ^= *r* ^A^, *p* ^B^ *, r* ^B/A ^= *r* ^B/a^	774.29	7.71	0.02	8	758.29
Dingo—Red‐legged pademelon					
psi^A^ (gc), psi^B/A ^= psi^B/a^ (gc), *p* ^A ^= *r* ^A^, *p* ^B^, *r* ^B/A ^= *r* ^B/a^	1,758.81	0.00	0.50	6	1,746.81
psi^A^ (gc), psi^B/A ^= psi^B/a^ (gc), *p* ^A^, *p* ^B^, *r* ^A^, *r* ^B/A ^= *r* ^B/a^	1,760.09	1.28	0.26	7	1,746.09
Dingo—Red‐necked pademelon					
psi^A^, psi^B/A ^= psi^B/a^, *p* ^A ^= *r* ^A^, *p* ^B^, *r* ^B/A ^= *r* ^B/a^	977.65	0.00	1.00	5	967.65
psi^A^, psi^B/A ^= psi^B/a^, *p* ^A ^= *r* ^A^, *p* ^B^, *r* ^B/A^, *r* ^B/a^	979.04	1.39	0.50	6	967.04
Dingo—Bandicoots					
psi^A^(gc), psi^B/A ^= psi^B/a^(gc), *p* ^A^, *r* ^A^, *p* ^B^, *r* ^B/A ^= *r* ^B/a^	1,259.11	0.00	1.00	8	1,243.11
psi^A^(gc), psi^B/A ^= psi^B/a^(gc), *p* ^A^, *p* ^B^, *r* ^A^, *r* ^B/A^, *r* ^B/a^	1,260.91	1.80	0.41	9	1,242.91
Dingo—Feral cat					
psi^A^(gc), psi^B/A ^= psi^B/a^, *p* ^A ^= *r* ^A^, *p* ^B^, *r* ^B/A^, *r* ^B/a^	848.79	0.00	1.00	7	834.79
psi^A^(gc), psi^B/A ^= psi^B/a^, *p* ^A^, *p* ^B^, *r* ^A^, *r* ^B/A^, *r* ^B/a^	850.41	1.62	0.44	8	834.41
Feral cat—Long‐nosed potoroo					
psi^A^, psi^B/A ^= psi^B/a^ (gc), *p* ^A ^= *r* ^A^, *p* ^B^, *r* ^B/A^, *r* ^B/a^	735.10	0.00	1.00	7	721.10
psi^A^, psi^B/A ^= psi^B/a^ (gc), *p* ^A^, *r* ^A^, *p* ^B^, *r* ^B/A ^= *r* ^B/a^	760.16	25.06	0.00	7	746.86
Feral cat—Red‐legged pademelon					
psi^A^, psi^B/A^, psi^B/a^, *p* ^A^, *p* ^B^, *r* ^A^, *r* ^B/A ^= *r* ^B/a^	1,438.32	0.00	1.00	7	1,424.32
psi^A^, psi^B/A^, psi^B/a^, *p* ^A^, *p* ^B^, *r* ^A^, *r* ^B/A^, *r* ^B/a^	1,440.32	2.00	0.37	8	1,424.32
psi^A^, psi^B/A^, psi^B/a^, *p* ^A ^= *r* ^A^, *p* ^B ^= *r* ^B/a^, *r* ^B/A^	1,444.01	5.69	0.06	6	1,432.01
Feral cat—Red‐necked pademelon					
psi^A^, psi^B/A ^= psi^B/a^, *p* ^A^, *p* ^B^, *r* ^A^, *r* ^B/A ^= *r* ^B/a^	845.32	0.00	1.00	6	833.32
psi^A^, psi^B/A ^= psi^B/a^, *p* ^A^, *p* ^B^, *r* ^A^, *r* ^B/A^, *r* ^B/a^	846.22	0.90	0.64	7	832.22
psi^A^, psi^B/A ^= psi^B/a^, *p* ^A^, *r* ^A^, p^B ^= *r* ^B/A ^= *r* ^B/a^	847.21	1.89	0.39	5	837.21
Feral cat—Bandicoots					
psi^A^, psi^B/A ^= psi^B/a^, *p* ^A^, *r* ^A^, *p* ^B ^= *r* ^B/A ^= *r* ^B/a^	1,027.72	0.00	1.00	5	1,017.72
psi^A^, psi^B/A ^= psi^B/a^, *p* ^A ^= *r* ^A^, *p* ^B ^= *r* ^B/a^, *r* ^B/A^	1,028.77	1.05	0.59	5	1,018.77
psi^A^, psi^B/A ^= psi^B/a^, *p* ^A^, *p* ^B^, *r* ^A^, =*r* ^B/a^, *r* ^B/A^	1,029.13	1.41	0.49	6	1,017.13
psi^A^, psi^B/A ^= psi^B/a^, *p* ^A^, *r* ^A^, *p* ^B ^= *r* ^B/a^, *r* ^B/A^	1,029.31	1.59	0.45	6	1,017.31
psi^A^, psi^B/A ^= psi^B/a^, *p* ^A ^= *r* ^A^, *p* ^B^, *r* ^B/a^, *r* ^B/A^	1,029.56	1.84	0.40	6	1,017.56

Note

Top 2 models or those <2∆AIC of the top model. Species A is the first listed species and species B the second listed. psi^A ^= probability of occupancy of species A, psi^B/A^ = probability of occupancy for species B, given species A is present, psi^B/a ^= probability of occupancy for species B, given species A is absent, *p* ^A ^= probability of detecting species A, given only species A is present, *p* ^B ^= probability of detecting species B, given only species B is present, *r* ^A ^= probability of detecting species A, given both species are present, *r* ^B/A ^= probability of detecting species B, given both species are present and species A is also detected, *r* ^B/a ^= probability of detecting species B, given both species are present and species A is not detected.

The article "Habitat and introduced predators influence the occupancy of small threatened macropods in subtropical Australia" was published in 2019. Journal: Ecol Evol.

Abbreviation: gc, ground cover.

#### 3.2.3 Dingo and red‐necked pademelon

The model with the best support estimated the probability of occupancy of the red‐necked pademelon as equal whether the dingo was present or not (psi^B/A ^= psi^B/a^ = 0.27 ± 0.05). Occupancy of the dingo was estimated as psi^A^ = 0.33 ± 0.06. The detection probability of the red‐necked pademelon was equal when dingoes were present and detected, and present and not detected (*p* ^B/A ^= *p* ^B/a ^= 0.38 ± 0.07) which was higher than detection when dingoes were absent (*p* ^B ^= 0.12 ± 0.04). Detection of the dingo was equal whether the red‐necked pademelon was detected or not (*p* ^A ^= *r* ^A^ = 0.14 ± 0.03). The estimates of phi and delta were both 1.0, suggesting one species did not influence the other.

#### 3.2.4 Dingo and bandicoots

The model with the best support estimated the probability of occupancy of bandicoots as equal whether the dingo was present or not (Table 4). Furthermore, occupancy of both was influenced by the habitat variable ground cover (Figure 4). The probability of detecting bandicoots was equal when dingoes were present and detected, and present and not detected (*r* ^B/A ^= *r* ^B/a ^= 0.13 ± 0.04) which was lower than their probability of detection when dingoes were absent (*p* ^B^ = 0.24 ± 0.03). Detection of the dingo was higher when bandicoots were present (*r* ^A ^= 0.19 ± 0.04) compared to when bandicoots were absent (*p* ^A^ = 0.06 ± 0.04). The estimates of phi and delta were both 1.0, suggesting one species did not influence the other.

#### 3.2.5 Dingo and feral cat

The model with the best support estimated the probability of occupancy for the feral cat as the same whether the dingo was present or not (psi^BA^ = psi^B/a^ = 0.46 ± 0.07). Dingo occupancy was most influenced by ground cover (0%–30% = 0.41 ± 0.08; 31%–50% = 0.31 ± 0.06; 51%–70% = 0.22 ± 0.06; 71%–100% 0.15 ± 0.07) (Table 4). Detection of feral cats was equivalent at sites when only feral cats were detected (*P* ^B ^= 0.12 ± 0.03) and sites where dingoes were present and detected (*r* ^B/A ^= 0.15 ± 0.08). However, the detection probability was lower when dingoes were present and not detected (*r* ^B/a ^= 0.02 ± 0.02). The estimate of phi was 1 suggesting that the occupancy of one species did not influence the occupancy of the other. The estimate of delta was 3.29 (95%CI = 0.76–5.8) suggesting the detection of one species was influential over the other. However, the 95% CI overlapped 1.0 indicating a variable response.

The article "Habitat and introduced predators influence the occupancy of small threatened macropods in subtropical Australia" was published in 2019. Journal: Ecol Evol.

#### 3.2.6 Feral cat and long‐nosed potoroo

The model with the best support estimated the probability of occupancy of the potoroo as the same whether the feral cat was present or not with ground cover being influential over long‐nosed potoroos (psi^B/A ^= psi^B/a ^= 0%–30% = 0.22 ± 0.58; 31%–50% = 0.28 ± 0.06; 51%–70% = 0.37 ± 0.09; 71%–100% 0.46 ± 0.13) with feral cat probability of occupancy being psi^A ^= 0.38 ± 0.09 (Table 4). Detection of the long‐nosed potoroo was equivalent when feral cats were present but not detected (*r* ^B/a ^= 0.20 ± 0.08) compared to when feral cats were present and detected (*r* ^B/A ^=^ ^0.15 ± 0.10) and when feral cats were not present (*p* ^B ^= 0.18 ± 0.05). The estimate of phi was 1.0, suggesting that the occupancy of one species did not influence the other. The estimate of delta was 0.79 (95%CI = 0.22–1.76) suggesting a lower likelihood that feral cats and long‐nosed potoroos were detected together but the 95%CI overlapped 1.0 indicating a variable response.

#### 3.2.7 Feral cat and red‐legged pademelon

The model with the best support estimated the probability of occupancy for the red‐legged pademelon as different when feral cats were present (psi^B/A ^= 0.75 ± 0.08) compared to when feral cats were absent (psi^B/a ^= 0.16 ± 0.09) (Figure 4, Table 4). Feral cat probability of occupancy was 0.78 ± 0.07. No habitat variables were influential over either species probability of occupancy. Detection of the red‐legged pademelon was higher when feral cats were absent (*p* ^B ^= 0.95 ± 0.11) compared to when feral cats were present and detected, and present and not detected (*r* ^B/A ^= *r* ^B/a ^= 0.28 ± 0.03). Feral cats had a higher detection probability when red‐legged pademelons were absent (*p* ^A ^= 0.11 ± 0.04) compared to when red‐legged pademelons were present (*r* ^A ^= 0.04 ± 0.01). The estimate of phi was 1.21 ± 0.11, 95%CI = 0.98–1.43 suggesting that the occupancy of feral cats was influential over the occupancy of red‐legged pademelons but variable. The modeling revealed a delta of 1.0 suggesting the detection of one species was not influential over the other.

#### 3.2.8 Feral cat and red‐necked pademelon

The model with the best support estimated the probability of occupancy for the red‐necked pademelon as the same when feral cats were present or not (psi^B/A ^= psi^B/a ^= 0.30 ± 0.07) with the probability of occupancy for feral cats being 0.46 ± 0.10. No habitat variables were influential over red‐necked pademelon or feral cat probability of occupancy in the top model. Detection of the red‐necked pademelon was lower when feral cats were absent (*p* ^B ^= 0.09 ± 0.06) compared to when feral cats where present and detected or not detected (*r* ^B/A ^= *r* ^B/a ^= 0.33 ± 0.07). Feral cats had a higher detection probability when red‐necked pademelons were absent (*p* ^A ^= 0.12 ± 0.03) compared to when they were present (*r* ^A ^= 0.02 ± 0.01). The estimate of both phi and the detection interaction factor was 1.0, suggesting one species was not influential over the occupancy or detection of the other.

The article "Habitat and introduced predators influence the occupancy of small threatened macropods in subtropical Australia" was published in 2019. Journal: Ecol Evol.

#### 3.2.9 Feral cat and bandicoots

The model with the best support estimated the probability of occupancy of bandicoots as equal when the feral cat was present or absent (psi^B/A ^= psi^B/a ^= 0.40 ± 0.05) (Table 4). The probability of detecting bandicoots was equal when feral cats were absent, present and detected and present and not detected (*p* ^B ^= *r* ^B/A ^= *r* ^B/a ^= 0.21 ± 0.03). The detection of feral cats was slightly lower when bandicoots were absent (*p* ^A ^= 0.07 ± 0.03) compared to when bandicoots were present (*r* ^A ^= 0.14 ± 0.04). The estimates of phi and delta were both 1.0, suggesting that neither of these species were influential over each other.

## 4 DISCUSSION

The landscape of fear hypothesis proposes that habitat used by prey species comprises high to low risk patches as determined by the presence and ubiquity of predators within an ecosystem (Laundré et al., 2014; Shrader et al., 2008). This results in a landscape of risky versus safe areas for prey species that can be reflected in the quality and availability of habitat (Laundré et al., 2014). Our study landscape comprised a gradient of habitat quality and availability where the dingo and feral cat were widespread and the red fox was sparse. Applying the LoF, we hypothesized that occupancy of smaller prey species (potoroo and bandicoot) would be higher in structurally complex habitats where they could avoid encounters with predators. Conversely, we predicted that larger cursorial prey species would be higher in structurally simplistic habitats because larger prey species (pademelons) escape predators by attempting to out run them. Our observations were broadly consistent with our habitat predictions though the direction of habitat influence varied among species. We also detected positive relationships between the dingo and long‐nosed potoroo, and the feral cat and red‐legged pademelon, suggesting either a targeting of prey by the predators or landscape factors that favored co‐occurrence.

The article "Habitat and introduced predators influence the occupancy of small threatened macropods in subtropical Australia" was published in 2019. Journal: Ecol Evol.

Whilst our results suggest that habitat selection for medium‐sized mammals may be consistent with the landscape of fear hypothesis, some shortcomings of our study were that: (a) our survey design deployed cameras in linear transects adjacent to roads and tracks rather than a grid layout which would have provided greater spatial coverage, (b) camera trapping with lures may draw animals away from their preferred microhabitats, (c) our camera trapping data were based on weekly records which may not describe interactions between predators and prey as well as an approach with a finer temporal resolution, and (d) our survey design used 500 m spacing between cameras to account for long‐nosed potoroo and red‐legged pademelon home ranges and thus were not intended to account for the much larger home ranges of predators that could move between sites. Therefore, occupancy for predators (dingoes and feral cats) may be better described as activity. However, we accounted for these short comings by: (a) utilizing a large spatial coverage of 298 sites in nine reserves across a landscape of 50 × 100 km, (b) conducting our surveys in 3‐week periods over 2 years, and (c) conducting surveys in the presence of just two broad vegetation types, and (d) capturing a gradient in occurrence of most species across our study landscape and restricting co‐occurrence modeling to conservation reserves where the two subject species were present.

### 4.1 Habitat and conservation reserves

Habitat selection may reflect a preference for foraging sites, for predator avoidance and in some cases a trade‐off between the two (Creel et al., 2005; Laundré, Hernández, & Altendorf, 2001). Smaller animals that are incapable of out running predators are likely to seek refuge in dense habitats to avoid detection and pursuit, particularly when rearing young (Signorell et al., 2010), whereas larger species that are capable of rapid movement have a higher chance of evading predation in more open habitats (Creel et al., 2005). Consistent with previous studies, we found that occupancy of the long‐nosed potoroo was influenced strongly by dense ground cover (Claridge & Barry, 2000; Norton et al., 2011) and occupancy of the red‐legged pademelon was strongly influenced by areas of open ground cover (Vernes, 1995). The long‐nosed potoroo's requirement for dense ground cover over other habitat variables may reflect a need for concealment from terrestrial predators, and habitat for diurnal nesting sites. In contrast, the red‐legged pademelon is a larger more mobile species capable of rapid movement and thus may have a preference toward more open habitats (which provide additional food rewards) and provide better opportunities to escape predators (Wahungu et al., 2001). Their ability to out‐run dingoes is suggested by many images from our cameras of pademelons displaying rump wounds which we presume are caused by dingoes giving chase to pademelons.

The article "Habitat and introduced predators influence the occupancy of small threatened macropods in subtropical Australia" was published in 2019. Journal: Ecol Evol.

We hypothesized that the threatened macropod species would occur in a subset of conservation reserves due to ongoing range contractions and loss of habitat connectivity within the landscape. The long‐nosed potoroo was only detected in five of the nine reserves and had much higher occupancy in the Border Ranges compared to the other reserves, perhaps reflecting an ongoing decline or vulnerability by this species. The absence of long‐nosed potoroos from Yabbra, Koreelah, Mebbin, and Mt Jerusalem may reflect past land use (logging) as all of these reserves were previously selectively cleared. All reserves where potoroos were present and detected included large areas of subtropical rainforest which were not as intensively logged compared to eucalypt forest. Subtropical rainforest may have provided important refugia.

The black‐striped wallaby showed the most extreme distributional pattern, being limited to just Richmond Range, but with too few records for analysis. The red‐legged pademelon was distributed throughout all conservation reserves, but it had high occupancy in some reserves (Richmond Range, Mebbin, Nightcap, Toonumbar, and Yabbra) and low occupancy in others (Border Ranges, Koreelah, Tooloom, and Mt Jerusalem).

Previous studies have shown that potoroos occupy a broad‐range of vegetation communities across their distribution. Our study confirms this but is the first to identify that subtropical rainforest provides important habitat. We confirm that structural complexity of understory vegetation is critical to this species. Claridge, Seebeck, and Rose (2007) identified coastal sandy wet heathlands, moist inland woodlands and forests on plateaux and their associated slopes and gullies to be important for potoroos across eastern Australia. Norton et al., (2011) found that potoroos showed a preference for dry forest when compared to heath and wet forest. On the coastal plains of subtropical Australia, potoroo habitat includes heathlands, heathy woodlands, open sclerophyll forest, and swamp sclerophyll forest (Andren et al., 2013), however, subtropical rainforest has not been identified as an important habitat for potoroos. We presume that this was because the majority of lowland subtropical rainforest in this study area (north‐east NSW), and more generally, eastern Australia had been destroyed by land clearing (Keith, 2004; Parkes et al., 2012).

Occupancy of red‐legged pademelons was highest at sites with open ground cover and least at sites with dense ground cover. Our findings are consistent with the findings of Vernes (1995) that red‐legged pademelons forage primarily in open habitat. In addition to open habitats, previous studies have found that red‐legged pademelons also require dense understorey vegetation, such as rainforests, wet sclerophyll forests, and dry vine thickets (Johnson & Vernes, 1995).

The article "Habitat and introduced predators influence the occupancy of small threatened macropods in subtropical Australia" was published in 2019. Journal: Ecol Evol.

### 4.2 Predators and co‐occurrence patterns

We hypothesized that dingoes and feral cats would be widespread throughout our study area and that they would have a positive relationship with their medium‐sized mammal prey as a result of seeking out habitats where prey occur. We also predicted that the association between dingoes and feral cats would be neutral. Our observations were largely consistent with these predictions. However, we also identified that the dingo had very high occupancy in Richmond Range NP and feral cats had extremely high occupancy in the Border Ranges NP, a rainforest reserve. The red fox was only detected at six of the 298 sites (naïve *ψ* = 0.02) which contrasted with the occupancy of dingoes and feral cats (naïve *ψ* = 0.17 and 0.13, respectively). This result was remarkably consistent with older studies in adjacent regions (Catling & Burt, 1997) and perhaps was consistent with the hypothesis that dingoes may exert control over this mesopredator (Johnson & VanDerWal, 2009; Letnic et al., 2011).

Occupancy of dingoes was influenced by ground cover with the highest probability of occupancy at sites with open ground cover. No other habitat variables (canopy, shrub cover, or vegetation type) were influential on dingo occupancy. Occupancy of dingoes had a positive relationship with the long‐nosed potoroo with the species interaction highest in areas of open ground cover. This suggests that areas of open ground cover habitat provide dingoes with opportunities to exploit potoroos as prey. The dingo is a broad‐ranging generalist carnivore that will consume a variety of prey based on their availability (Newsome & Coman, 1989). Medium‐sized mammals make up the majority of the dingo diet in subtropical Australia (Doherty et al., 2018). Previous studies of dingo diet in Richmond Range found that red‐necked pademelons make up a large portion of their diet (Barker et al., 1994; Glen, Fay, & Dickman, 2006); however, this study did not detect potoroos in dingo scats.

Biannual (spring and autumn) lethal baiting with 1,080 took place in five of our nine conservation reserves during this study, however, this did not have an influence on dingo occupancy. This is consistent with the findings of some studies (see Allen et al., 2015) however, inconsistent with others (Fleming, 1996). There are a number of possibilities that may explain the weak effect of baiting on dingo occupancy; (a) the effectiveness of baiting programs are greatly dependent on the intensity of the baiting regime, (b) our study landscape is dynamic and provides continuous habitat for large ranging predators, with adjacent areas of habitat available where dingoes can move between and re‐occupy our study area if mortality occurs as a result of baiting, (c) dingoes have large home ranges and are able to move between camera monitoring sites (Claridge, Mills, Hunt, Jenkins, & Bean, 2009), and (d) the short‐term nature of this study does not account for longer seasonal and temporal patterns of dingo movement and habitat use (Ballard, Fleming, & Meek, 2018). Further detailed studies are required to determine the effect of baiting on dingo populations in our landscape.

The article "Habitat and introduced predators influence the occupancy of small threatened macropods in subtropical Australia" was published in 2019. Journal: Ecol Evol.

The feral cat was not influenced by any habitat covariates, occurring across both vegetation types and a range of habitat attributes. Our results showed a positive relationship between occupancy of feral cats and red‐legged pademelons. Although it is widely accepted that birds, reptiles and small mammals are the preferred prey of feral cats in densely forested habitats, feral cats also prey upon medium‐sized mammals (Doherty et al., 2015; Radford et al., 2018). Fancourt (2015) documented a cat killing an adult female Tasmanian pademelon (*Thylogale billardierii*) weighing approximately 4 kg. Fancourt (2015) also found a correlation between the decline in Tasmanian bettongs (*Bettongia gaimardi*) and cat activity, and implicated the feral cat as being the driver of this decline. In our study, the detection of the red‐legged pademelon was much higher (0.95) when the feral cat was absent compared to when it was present and detected or not (0.28). This finding is consistent with the idea that red‐legged pademelons are more active when feral cats are absent. It is suspected that the period when medium‐sized mammals are most vulnerable to cat predation is during the “young‐at‐foot‐phase.” Our study did not model young‐at‐foot detections of medium‐sized mammals due to limited observations. Continuous monitoring may improve young‐at‐foot detections and allow modeling to infer further detail on the relationship between feral cats and medium‐ sized mammals in our study area.

We predicted that the dingo and feral cat would have a neutral occupancy relationship. Our data suggest that feral cat occupancy was the same whether the dingo was present or absent which supports our prediction. Very few studies have detected a relationship between dingoes and feral cats (see Allen et al., 2015). Wang and Fisher (2012) observed a fine scale temporal segregation between feral cats and dingoes in central Queensland, as a function of the season (December–March wet period) when dingo activity increased however, the spatial activity of feral cats and dingoes was highly overlapping suggesting that both predators were selecting habitats with similar qualities. Although we did not detect a spatial relationship between dingoes and feral cats, the detection of the feral cat was marginally lower when the dingo was present and not detected compared to when the dingo was present and detected with the detection interaction factor being very high, which suggests that there may be a temporal effect of dingoes on feral cat detectability. However, given the variability of the detection interaction confidence intervals, this conclusion should be treated with caution. Although predation of feral cats by dingoes has been observed in arid regions (Moseby, Neilly, Read, & Crisp, 2012), given the spatial distribution of dingoes and feral cats across our study landscape, we suspect that feral cats are able to evade dingo predation in complex mesic ecosystems.

The article "Habitat and introduced predators influence the occupancy of small threatened macropods in subtropical Australia" was published in 2019. Journal: Ecol Evol.

### 4.3 Significance and broader implications of the study

The structure and quality of habitat and its availability can be a strong factor determining the occurrence and movement of ground‐dwelling mammals (Law & Dickman, 1998), particularly in areas where introduced predators are present (Hradsky et al., 2017; Robinson et al., 2013). We found that habitat structure was influential over the occupancy of two threatened macropods, the long‐nosed potoroo and the red‐legged pademelon in landscapes where the dingo and feral cat were present. These findings have implications for the management of habitat for these species, particularly when considering actions that instigate change in habitat structure, for example, fire and environmental weed management. Considerations should be given to the spatial coverage of actions likely to simplify understory habitat where potoroos and red‐legged pademelons occur so as to allow for adequate refugia in the presence of introduced predators. Whilst this study has revealed some important relationships concerning habitat preference and potential predator–prey interactions, these relationships may be revealed in greater detail through a survey design that is focussed on fewer reserves to provide a higher spatial and temporal resolution where the threatened macropods are most abundant.

## CONFLICT OF INTEREST

None declared.

## AUTHOR CONTRIBUTIONS

DM executed field work, processed images, collated data, analysed data and wrote the manuscript; RG designed the study, analysed the data, assisted in writting the manuscript and gave editorial advise; JL executed field work and processed images; ML assisted in designing the study and gave editorial advise.

The article "Habitat and introduced predators influence the occupancy of small threatened macropods in subtropical Australia" was published in 2019. Journal: Ecol Evol.

## Data Availability

Data used for analysis in this study are accessible at Dryad (https://osf.io/vkyt5/files).
